This article has been retracted.

# COVID-19 Detection Based on Lung Ct Scan Using Deep Learning Techniques

**DOI:** 10.1155/2022/7672196

**Published:** 2022-02-01

**Authors:** S. V. Kogilavani, J. Prabhu, R. Sandhiya, M. Sandeep Kumar, UmaShankar Subramaniam, Alagar Karthick, M. Muhibbullah, Sharmila Banu Sheik Imam

**Affiliations:** ^1^. Department of Computer Science and Engineering, Kongu Engineering College, Perundurai, Erode 638060, Tamil Nadu, India; ^2^School of Information Technology and Engineering, Vellore Institute of Technology, Vellore, Tamil Nadu, India; ^3^Renewable Energy Lab, College of Engineering, Prince Sultan University, Riyadh, Saudi Arabia 11586; ^4^Department of Energy and Environmental Engineering, Saveetha School of Engineering, Saveetha Institute of Medical and Technical Sciences, Saveetha University, Saveetha Nagar, Thandalam, Chennai-602105, Tamilnadu, India; ^5^Renewable Energy Lab, Department of Electrical and Electronics Engineering, KPR Institute of Engineering and Technology, Coimbatore, 641407 Tamilnadu, India; ^6^Department of Electrical and Electronic Engineering, Bangladesh University, Dhaka 1207, Bangladesh; ^7^College of Computer Science & Information Technology (CCSIT), King Faisal University, Alahsa, Saudi Arabia 31982

## Abstract

SARS-CoV-2 is a novel virus, responsible for causing the COVID-19 pandemic that has emerged as a pandemic in recent years. Humans are becoming infected with the virus. In 2019, the city of Wuhan reported the first-ever incidence of COVID-19. COVID-19 infected people have symptoms that are related to pneumonia, and the virus affects the body's respiratory organs, making breathing difficult. A real-time reverse transcriptase-polymerase chain reaction (RT-PCR) kit is used to diagnose the disease. Due to a shortage of kits, suspected patients cannot be treated promptly, resulting in disease spread. To develop an alternative, radiologists looked at the changes in radiological imaging, like CT scans, that produce comprehensive pictures of the body of excellent quality. The suspected patient's computed tomography (CT) scan is used to distinguish between a healthy individual and a COVID-19 patient using deep learning algorithms. A lot of deep learning methods have been proposed for COVID-19. The proposed work utilizes CNN architectures like VGG16, DeseNet121, MobileNet, NASNet, Xception, and EfficientNet. The dataset contains 3873 total CT scan images with “COVID” and “Non-COVID.” The dataset is divided into train, test, and validation. Accuracies obtained for VGG16 are 97.68%, DenseNet121 is 97.53%, MobileNet is 96.38%, NASNet is 89.51%, Xception is 92.47%, and EfficientNet is 80.19%, respectively. From the obtained analysis, the results show that the VGG16 architecture gives better accuracy compared to other architectures.

## 1. Introduction

COVID-19 is a disease, caused by a virus (SARS-CoV-2). Infections in the lungs can range from a simple cold to a life-threatening condition. Symptoms of the respiratory system often accompany infections caused by coronaviruses. Individuals may have minor, self-limiting illnesses with adverse effects like influenza on rare occasions. Fever, cough, and difficulty breathing are among the symptoms of respiratory issues, weariness, and a sore throat [1–3]. The use of X-rays and computed tomography scans is one of the fundamental approaches to diagnosing COVID-19. Chest imaging is a quick and efficient method suggested by medical health regulations, and it has been highlighted in several papers as the first instrument in epidemic screening. Different computer vision approaches are used, such as segmentation and classification. When a quick and straightforward method running on limited computing devices is needed, an automated technique that can provide fragmentation and measurement of the infection region of patients every three to five days and monitor the evolution of infected patients through CT scan imaging and clinical detection is required. COVID-19 is a difficult disease to diagnose, even for expert doctors [4, 5].

Many studies have been undertaken on the use of deep learning in the interpretation of radiological images. They have been undertaken to solve the constraints of COVID-19 medical techniques based on radiological images. The CNN architecture is the most effective approach for detecting it among the most significant deep learning algorithms. Data processing of deep learning algorithms, notably CNN, has received much interest.

In early 2020, the COVID-19 outbreak became a worldwide epidemic. The World Health Organization declared a significant international public health emergency, and the condition was considered a health emergency. Automatic detection of lung infections through CT scans provides an excellent opportunity to extend traditional healthcare methods to address COVID-19. But CT has many problems [1]. CNN is used to detect lung tumors, pneumonia, tuberculosis, emphysema, or other pleural diseases. The disadvantages of the CT system are as follows: because the contrast of the soft tissues is lower than that of the MRI, it is an X-ray Radiation exposure [6].

Using deep learning algorithms, the suspected patient's X-ray and CT scan can be distinguished between a healthy person and a COVID-19 patient. Deep learning models are employed in creating diagnosis systems for COVID-19. DenseNet121, VGG16, Xception, EfficientNet, and NASNet are the architectures employed, and multiclass classification is used. Positive individuals with COVID-19, regular patients, and other patients are also considered. Chest X-ray images indicate pneumonia, flu, and other chest-related disorders that belong in another category. VGG16 achieves 79.01% accuracy, EfficientNet achieves 93.48 accuracy, Xception achieves 88.03 accuracy, NASNet achieves 85.03 accuracy, and DenseNet121 achieves 89.96% accuracy [7].

For disease diagnosis, the algorithms presented include the DNN based on imaging features of fractals and the CNN that directly uses lung imaging. The suggested architecture of CNN, with higher accuracy of 93.2% and a sensitivity of 96.1%, outperforms the DNN technique with 83.4% precision and 86% sensitivity. A CNN architecture is offered during the segmentation phase to detect contaminated tissue in the lung pictures. The results show that this method can see almost 4,444 infected areas with an accuracy rate of 83.84%. And the finding is used to monitor and control the growth of the patient's protected area [8].

Preprocessing, dictionary building, and picture classification are the three critical stages of the classification approach based on features. In the suggested method, features are manually retrieved and passed to a classifier neural network than modern methods in an experimental environment. On three data sets, the technique has an accuracy of 96.1, 99.84, and 98%. These results are superior to those obtained using modern approaches. The SURF method is utilized to extract objects in a visual word bag. Because the SURF technique is dependent on gradients and the obtained solution is noise-sensitive, the offered approaches may misclassify the image if the image quality is inadequate. In this case, picking the proper pretreatment procedure can help you get better outcomes [9].

Using chest CT images, a new multicore deep neural network method is proposed to detect the COVID-19 disease, also known as COVID-19. This paper extracted the characteristics from lung CT images using a CNN. A predefined DenseNet201 CNN architecture based on transfer learning is employed for this purpose. The ELM method classifier depends on various activation algorithms that calculate the architecture's performance. According to the data, when applying the MKsELMDNN model, the accuracy score reached was 98.36% [10].

Machine learning techniques based on X-ray imaging are utilized as a decision support mechanism to assist radiologists in speeding up the diagnosis process. A critical review of 12 conventional CNN designs was first proposed for natural image processing to assist radiologists in distinguishing COVID-19 diseases from radiographic pictures of the chest. COVID-19 X-ray pictures were used, as well as a massive dataset of non-COVID viral illnesses, bacterial infections, and routine radiographs were also used. When trained on a tiny image dataset, a simple CNN design can outperform architectures like Xception and DenseNet. Finally, therapists should not examine CNN conclusions despite their excellent classification accuracy until they can visually analyze the region of the input image acquired by the CNN [11].

For automatic COVID-19 categorization, different deep learning methods by extracting their features were compared. MobileNet, ResNetV2, VGGNet, ResNet, InceptionV3, DenseNet, Xception, Inception, and NASNet have been selected from a vast list of convolutional neural networks to produce the most accurate feature, which is an integral part of learning. The collected features are fed into a series of machine learning classifiers to determine whether the subjects were COVID-19 cases or controls. This strategy achieved task-specific data preprocessing approaches to promote a robust generalization capacity for unknown data. The method's accuracy was tested using the publicly available COVID-19 dataset of chest X-ray and CT images. DenseNet121 achieved 99.5 percent accuracy with a bagging tree classifier, while ResNet50 achieved 50% accuracy [12].

Chest X-ray images have recently emerged as a promising option for COVID-19 screening when combined with current AI techniques, particularly DL algorithms. The classification of COVID-19 from standard cases was evaluated using eight architectures like AlexNet, GoogleNet, SqueezeNet, VGG-16, ResNet 50, MobileNet V2, ResNet 34, and Inception V3, respectively. The models have been evaluated on publicly accessible chest X-ray images, with ResNet-34 getting the best results, with an accuracy of 98.33 percent [13]. A CT scan involves slides of a hundred scans, and using such scans to diagnose COVID-19 can cause hospital delays. Artificial intelligence tools could help radiologists diagnose COVID-19 infections in these images more quickly and correctly. Using artificial intelligence, this study offers a technique for identifying COVID and non-COVID classes. The suggested AI method predicts COVID-19 in each 3D CT scan image using the ResNet-50 deep learning model. Using image-level predictions, an AI method detects COVID-19 in a 3D CT volume. With an accuracy of 96%, the suggested deep learning model detects the disease on CT images [14]. The ten possible best convolutional neural networks used to distinguish the infection are AlexNet, GoogleNet, VGG 19, ResNet 101, VGG 16, ResNet 50, MobileNet V2, ResNet 18, SqueezeNet, and xception. All of the networks performed well, except for ResNet-101 and Xception. For discriminating the disease, ResNet-101 had an accuracy of 99.4%, while Xception had an accuracy of 99.99%. ResNet-101 is a moderate model for identifying and detecting COVID-19 infections in radiology departments that may be used as a replacement [15].

DenseNet, InceptionV3, and Inception-ResNetV4 were recommended as three different models. In the investigation, chest X-ray radiographs were used to diagnose individuals with COVID-19 and pneumonia. Using 5-fold cross-validation, these three models create and evaluate ROC curve analyses and uncertainty matrices. The pretrained DenseNet architecture achieved an optimum classification efficiency of 92 percent in simulations, while the other two models, Inception V3 and Inception-ResNetV4, achieved 83.47 percent and 85.57 percent, respectively [16]. Radiological imaging using advanced artificial intelligence techniques can aid in precise disease detection and overcome the shortage of expert physicians in rural areas. This paper offers a new method for automated COVID-19 identification based on raw chest X-ray images. The suggested technique offers correct diagnostics for binary and multiclass classification in binary and multiclass environments. The model gives an accuracy of 98.08% for binary classes and 87.02% for the instance of multiclass [17]. The binary classification method was trained using 3,877 CT and X-ray images, including 1,917 COVID-19 patients. The binary classification had a 99.64% overall accuracy, 99.58% recall, 99.56% precision, 99.59% *F*1-score, and 100% ROC. Normal healthy people contain instances of 1917, normal healthy people contain instances of 1,960, and pneumonia contains 2200 instances. By using these instances, the classifier was tested on a total of 6,077 images for different classifications. The multiclass has a 99.87% ROC, 98.2% accuracy, 98.25% recall, 98.22% *F*1-score, 98.22% precision, and 98.22% precision [18]. The VGG16 and ResNet50 models are improved and optimized using augmentation of data and fine-tuning strategies. The model's resilience and effectiveness were also tested using stratified 5-fold cross-validation. It performs exceptionally well in binary classification, with an average accuracy rate of more than 99% in the VGG16 and ResNet50 model models. Using the architectures as baselines, the model achieves an overall classification accuracy of 86.74 percent in multiclass classification and 88.52 percent in single-class classification. Experiments have shown their model exceeds the competition, which is used automatically to detect COVID-19 in CT scans [19].

The Bat algorithm (BA) is a nature-inspired meta-heuristic algorithm commonly utilized to address universal management problems in the real world. While dealing with complicated real-world situations, one of the key obstacles the BA faces is its repeated entrapment in local optimization. The updated version of the Bat algorithm can also benefit medical image classification [20]. Since animal unstructured text data can be collected from Twitter, supervised machine learning algorithms such as deep neural networks can recognize online individuals suffering from depression [21]. Particle Swarm Optimization (PSO) is a swarm-based smart stochastic optimization approach inspired by the natural way bees swarm when looking for food. It is mainly used to solve multiple types of optimization issues. Particle swarm optimization methods are commonly used to diagnose diseases [22]. CNN is an effective tool for selecting the best features to improve prediction accuracy. The LSTM model conserves leading-up relevant information, which aids in extracting important context information at the beginning of a sentence. The CNN + LSTM framework for personality factor classification combines CNN and LSTM to help categorize input text into various personality qualities. The integrated framework is also used to detect psychopaths and gives the best accuracy of 91.67% for classification [23, 24].

The contribution of this research work is to

- Collect the COVID-19 sample dataset from Kaggle, containing 3873 CT scan images
- Preprocess the dataset to make all images of literature the same size
- The preprocessed dataset is split into training, validation, and test data
- The training dataset is fed into different CNN architectures like Xception, MobileNet, NASNet, DenseNet121, EfficientNet, and VGG16
- The trained models are validated using a validation dataset with 50 epochs
- Now the models are being tested by supplying test data

A real-time reverse transcriptase-polymerase chain reaction (RT-PCR) kit is used to diagnose the disease. Due to a shortage of kits, suspected patients cannot be treated promptly, resulting in disease spread. To develop an alternative, radiologists looked at the changes in radiological imaging, like CT scans, that produce comprehensive pictures of the body of excellent quality. The rest of this paper is formulated in the following way: the recent COVID-19 identification study results are presented in the literature review. The proposed system section discusses the detection of COVID-19. This section also gives a complete description of the classification models utilized in the proposed system. The steps involved in the architecture are described in the section on system architecture. The Results and Discussion section contains a complete analysis and comparison of the performance of the CNN models. Finally, a summary of the proposed work and future work is specified in the Conclusion section.

## 2. Materials and Method

### 2.1. Deep Learning Techniques

Artificial intelligence techniques that resemble how humans acquire knowledge and deep learning are similar to machine learning techniques. Data science, which covers statistics and predictive modeling, includes deep learning as a critical component. In deep understanding, a convolutional neural network is a kind of deep neural network used to analyze visual imagery. A deep learning method, CNN takes an input image and assigns weight to various objects in the picture, allowing it to differentiate between them. Because of its great accuracy, CNN is used to classify and identify images [25].

### 2.2. Classification

Deep learning architectures, namely, VGG16, DenseNet, MobileNet, Xception, EfficientNet, and NASNet, are used to classify the data. Transfer learning is used to train these models. Each model has been trained for a total of 50 epochs. A detailed explanation is given below.

### 2.3. Xception

The Xception network has replaced the Inception network. Extreme inception is often referred to as Xception. Instead of typical convolution layers, the Xception network uses depth-wise separable convolution layers. Xception includes mapping spatial and cross-channel correlations, which in CNN feature maps can be completely dissociated. The underlying Inception architecture survived longer than Xception. The 36 convolution layers in the Xception model can be separated into 14 different modules. After the first and last layers are removed, every layer has a continuous residual link around it. The input image is converted into spatial correlations within each output channel to obtain the cross-channel correlations in an input image. After that, a depth-wise 1 × 1 convolution method is performed. Instead of 3D maps, the relationships may be viewed as a 2D + 1D map. In Xception, the first step is to do a 2D space correlation, followed by 1D space correlations [7]. The architecture is illustrated in Figure 1.

### 2.4. VGG16

VGG16 is a CNN model, and the VGG created the model at Oxford University. The network's replacement, AlexNet, was founded in 2012. VGG16 has eight layers, three completely connected layers, five max-pooling layers, and one softmax layer, as illustrated in Figure 2. As part of the ImageNet competition, the architecture has been designed. The convolution blocks' width is set to a low integer. The width parameter is expanded by two after each max-pooling operation till it reaches 512. The VGG16 is given an image size of 224 × 224 pixels. Spatial padding was used to maintain the image's spatial resolution. The VGG16 network has been released as open-source so that similar operations can be carried out. The model may also be used for transfer learning because specific frameworks, like Keras, provide pretrained weights that can be utilized to construct custom models with minor alterations [7].

### 2.5. MobileNet

MobileNet uses Depthwise separable convolutions. While compared to a network with regular convolutions of the same depth in the nets, it substantially reduces the number of parameters. As a result, lightweight deep neural networks are created. Depthwise separable convolution layers are used to construct MobileNets. Each depth-wise detachable convolution layer comprises a depth-wise convolution layer and a pointwise convolution layer. A MobileNet contains 28 layers if depthwise and pointwise convolutions are counted separately, and the model is defined in Figure 3. The width multiplier hyperparameter can be adjusted to reduce the number of parameters in a conventional MobileNet to 4.2 million. The input image is 224 × 224 pixels in size [15].

### 2.6. NASNet

The Google ML team created the NAS Network. Reinforcement learning is used to build the network architecture. The network adjustment is made based on the changes in the effectiveness of the child block. The parental block evaluates the effectiveness of the children's block. RNN and CNN are the network's components. Various changes to the architecture were made to gain the optimum performance from the web, including weights, regularisation methods, layers, and optimizer functions. Reinforced evolutionary processes select the best candidates and choose the best cells by utilizing various NASNet variants like A, B, and C algorithms [26]. The model is illustrated in Figure 4.

Using tournament selection techniques, the cells with the weakest performance are eliminated. The performance of the cell structure is enhanced by improving the child's objective functions and carrying out reinforcement mutations. A block is considered the smallest element, and a cell combines several blocks. The search space of the network is factored into cells, which are then divided into blocks. The dataset type determines the number of cells and blocks, which is not fixed. Convolutions, pooling, mapping, and other operations are executed within a block. NASNet was one of the methods used for identifying infected and not-infected patients because of its transferable learning methodology. With its minimal network design, it offers more possibilities [27].

### 2.7. DenseNet121

DenseNet is a densely connected neural network, a different technique to increase the extent of deep convolutional networks without experiencing problems like expanding gradients and disappearing gradients. Each layer connects directly with other layers where the maximum amount of information and gradient flow is passed. With this, the issues are solved. The objective is to focus on feature reuse rather than relying on large, deep, or broad CNN architectures for symbolic power. Compared to conventional CNN, DenseNets require fewer or equal numbers of nodes. Because the feature maps are not learned in DenseNets, and the parameters are not needed. Several ResNets versions have scarcely contributed, and those layers can be removed, and the model is defined in Figure 5.

DenseNet layers add only a few significant features, and the layers are narrow with only a few other filters. The issue emerges when training the data because deep neural networks incorporate information flow and gradients. DenseNets solves these issues by directly accessing the actual input's gradients and transfer functions. Dense Net's network design gets more hierarchical as feature translation from the (*i* − 1)^th^ level becomes the intake to the *p*^ith^ layer. The DenseNet is a generally applicable network since the input to the width layer can originate from any level (*i* − 1), (*i* − 2), or even (*i* − *n*) (where *n* must be less than the number of layers total). The network is normalized using a batch normalization phase, which reduces the actual error between the data and examines substantial variation [28].

### 2.8. EfficientNet

The scaling of the model is one of the most important considerations when utilizing CNNs. Increasing the model's depth improves the system's performance. On the other hand, selecting the model's depth is a challenging issue requiring a human hit-or-miss approach to choosing a better-performing model. MBConv is the core component of the EfficientNet models. A squeeze-and-excitation optimization block has been added to this block. The MBConv block in MobileNet V2 works similarly to the inverted residual blocks. To decrease the number of channels in the output, 3 × 3 depth-wise and pointwise convolutions are utilized to build a direct link between the start and finish of a convolutional block to reduce the number of channels in the output feature maps. The small layers are connected with low computational complexity, whereas the broader levels are associated with hidden neurons. The model's size and the number of functions in the structure are reduced by this architecture, which is illustrated in Figure 6. In this work, EfficientNetB6 is used to classify COVID-19 patients and healthy people.

### 2.9. Proposed System Architecture

Chest tomography CT scan images are given as the input. The process is illustrated in Figure 7. CT images are preprocessed. The image must fit the network's input size to train it and generate predictions on the data. The data is rescaled to check the network's input size. In the proposed system, the input image size is 224 × 224. So, the data is rescaled according to the input size.

CNN architectures like VGG16, MobileNet, DenseNet121, Xception, EfficientNet, and NASNet are performed to detect COVID-19. Data augmentation such as cropping and horizontal flipping generally produces new images by zooming in and out based on the input parameters given in Table 1. The number of training examples used in one iteration is referred to as the “batch size.” For all models, a batch size of 16 is chosen. Optimizers are algorithms used to change attributes of neural networks, such as weight and learning rate, to reduce losses. The Adam optimizer is used for optimization.

To reduce the nonlinearity in the output of a neuron, certain activation functions are used. The output layer's activation function determines the kind of predictions the model can make. In the proposed system, the softmax function is used as the activation function for all the models. Softmax is used in the last layer, the output layer, to predict a multinomial probability distribution. “Loss” is the network's prediction error, and the “loss function” is the method used to calculate the error. And the loss function also calculates gradients. Gradients are used to update the weights of the neural network. In binary classification tasks, binary cross-entropy compares predicted probability to actual class output, which might be either 0 or 1.

Image augmentation is expanding the available dataset for training the model. The dataset is divided into training, validation, and testing. The collection of samples used to learn how to suit the parameters is referred to as training. Validation is a collection of examples used to fine-tune a classifier's parameters. The data is trained and validated for 50 epochs, and the class probability of the images is then generated. The results were calculated by evaluating the performance measures such as accuracy, precision, recall, and *F*-score.

## 3. Performance Evaluation Measures

### 3.1. Dataset

The dataset collection includes lung CT scan images. A CT scan utilizes advanced X-ray technology to diagnose sensitive internal organs carefully. The dataset was taken from Kaggle and consisted of 3873 images. COVID and non-COVID are the two categories into which the data is divided. The COVID class includes CT scan images of COVID patients, while the non-COVID class includes healthy individuals. There are 1958 CT scan images in the COVID class and 1915 CT scan images in the non-COVID class. The model is trained on 70% of lung CT scans, validated on 15% of lung CT scans, and tested on 15%. These are illustrated in Table 2.

### 3.2. Preprocessing

A squared image with a predetermined aspect ratio is scaled to have roughly the same height and width. The image filtering preprocessing technique is used to filter the size of all input samples. In the proposed system, the images are rescaled to 224 × 224.

### 3.3. Image Augmentation

It is the process of expanding the existing dataset for training the model. Existing data is altered using generative adversarial networks (GAN) augmentation techniques to generate new images. GAN consists of two neural models, and the goal of the method is to learn from the training data and develop new data with the same characteristics as the training data. The description of the augmented dataset is illustrated in Table 3.

### 3.4. Performance Measures

There are several methods to evaluate a model's performance. Accuracy, precision, recall, and *F*-score are the measures considered to estimate chest CT scan images. In the general confusion, a matrix is represented as in Table 4.

Precision—precision is defined as the ratio of correctly predicted positive cases, given in the following equation.

(1) $$\begin{array}{c} \text{Precision}=\frac{\text{TP}}{\text{TP}+\text{FP}}. \end{array}$$

Recall—the ratio of accurately detected positive cases is the recall given in the following equation.

(2) $$\begin{array}{c} \text{Recall}=\frac{\text{TP}}{\text{TP}+\text{FN}}. \end{array}$$

*F*1-score—the *F*1-score is the harmonic mean of precision and recall given in the following equation.

(3) $$\begin{array}{c} F1\text{ score}=2\text{ x}\frac{\text{ Precision x Recall}}{\text{Precision}+\text{Recall}}. \end{array}$$

Accuracy: the percentage of correct predictions among the total number of predictions is called accuracy, specified in equation 4.

(4) $$\begin{array}{c} \text{Accuracy}=\frac{\text{TP}+\text{TN}}{\text{TP}+\text{FP}+\text{TN}+\text{FN}}. \end{array}$$

Precision, recall, *F*1-score, and support for the COVID class are illustrated in Table 5, and the non-COVID class is represented in Table 6.

From Table 5 and Table 6, it is clear that VGG16, with fewer convolution layers, could achieve the highest precision and *F*1-score than other models.

In practical implementation, the CNN models like Xception, MobileNet, DenseNet, NASNet, and EfficientNet have many more hyperparameters than the VGG16 model. Instead of having many hyperparameters, the VGG16 model supports 16 layers and focuses on the convolution layers of 3 × 3 filters in stride one and padding along with Max-pooling layers of 2x2 filters in stride 2. So the *F*1 score of VGG 16 performs better for both COVID and non-COVID classes compared to other CNN models[29 - 32].

## 4. Results and Discussion

The confusion matrix that lists the number of correct and wrong classification model predictions was also calculated. The confusion matrix obtained for all CNN models is illustrated in Figure 8.

By the analysis, VGG16 gives better results as the number of parameters trained in VGG16 is less, and it takes less time to train the samples. So, it is better than other CNN models.

The examination of the epoch versus loss and epoch versus accuracy in the suggested model is shown by graphs. The loss gained after each epoch is represented in the epoch versus loss graph. As the number of epochs increases, the loss values are reduced, as shown in Figure 9.

The epoch is the number of times the data has been cycled over. The error over the training set, usually in terms of regression or classification, is called loss. Increasing the number of epochs, on the other hand, improves the model's accuracy, which is shown in Figure 10. This shows that the model is effectively learning the provided input with each epoch.

Table 7 shows the difference between the accuracy obtained from the existing system and the proposed system. The results show that the deep learning CNN models give better accuracies for lung CT scan images when compared to the accuracies of lung X-ray images as specified in [7].

The accuracies attained for all CNN models are shown in Figure 11. The VGG16 model has been trained with 138 million parameters, which performs better than other CNN models. The 138 billion parameters available in VGG16 make this model a slower one, but this model is the best one to produce better accuracy. The VGG16 model gives an accuracy of 97%, the MobileNet model gives an accuracy of 96%, the Xception model gives an accuracy of 92%, the DenseNet121 model gives an accuracy of 97%, NASNet gives an accuracy of 89%, and EfficientNet gives an accuracy of 89%.

## 5. Conclusion

By analyzing CT scan images, the paper identifies widespread and best deep learning architectures to identify COVID-19 in suspected patients. Deep learning methods have been proposed to provide efficient results by evaluating ideas to detect the existence of COVID in an individual. High-performance deep learning architectures like VGG16, DenseNet, MobileNet, Xception, NASNet, and EfficientNet are used in this proposed work. Since the CT scan images collected by Kaggle contain fewer images, data augmentation is performed to get more pictures. The models performed well by applying preprocessing to the samples and performing CNN architectures on the training and validation datasets. The models classify COVID and non-COVID images, and their accuracy is tested using a test dataset and gives expected accuracy for all models. The model's performance is evaluated using performance measures like precision, recall, and *F*1-score. The highest accuracy acquired among all the models is VGG16, at 97.68%. Hence, the proposed system identifies the VGG16 model as the best model to classify the given CT scan images into COVID and non-COVID. But the limitation of the proposed work is that it does not identify COVID-affected areas in the lungs. A further enhancement is required to detect the affected areas in the lungs by considering a large dataset and applying other preprocessing techniques and pretrained models in transfer learning to improve the accuracy of the proposed CNN models. Future work may also investigate yolo architecture to achieve better accuracy.

## Figures and Tables

**Figure 1:** Xception architecture.

**Figure 2:** VGG16 architecture.

**Figure 3:** MobileNet architecture.

**Figure 4:** NASNet architecture.

**Figure 5:** DenseNet121 architecture.

**Figure 6:** Efficient net architecture.

**Figure 7:** Proposed system architecture.

**Figure 8:** Confusion matrix of CNN models.

**Figure 9:** Epochs versus loss graph for all CNN models.

**Figure 10:** Epochs versus accuracy graph for all CNN models.

**Figure 11:** Accuracies obtained for all CNN models.

**Table 1:** Parameters for training the models.

Performance measures	VGG16	DenseNet121	MobileNet	Xception	NASNet	EfficientNet
Batch size	16	16	16	16	16	16
Image dimension	224 × 224	224 × 224	224 × 224	224 × 224	224 × 224	224 × 224
Optimizer	Adam	Adam	Adam	Adam	Adam	Adam
Activation function	Softmax	Softmax	Softmax	Softmax	Softmax	Softmax
Loss function	Binary cross-entropy	Binary cross-entropy	Binary cross-entropy	Binary cross-entropy	Binary cross-entropy	Binary cross-entropy

**Table 2:** Kaggle dataset description.

Dataset	COVID	Non-COVID
Training	930	915
Validation	156	164
Test	166	150
Total	1252	1229

**Table 3:** Data augmentation dataset description.

Dataset	COVID	Non-COVID	Total
Training	1257	1234	2491
Validation	345	346	691
Test	356	335	691
Total	1958	1915	3873

**Table 4:** Confusion matrix representation.

	Predicted	
Actual	Yes	No
Yes	TP	TN
No	FN	FP

Where TP denotes “True Positive,” TN denotes “True Negative,” FN represents “False Negative,” and FP represents “False Positive”.

**Table 5:** Comparison of various evaluation measures for COVID class.

Performance measure	VGG16	DenseNet121	MobileNet	Xception	NASNet	EfficientNet
Precision	1.00	0.96	0.99	0.90	0.96	0.91
Recall	0.96	0.99	0.94	0.96	0.83	0.46
*F*1-score	0.98	0.98	0.96	0.93	0.89	0.61
Support	357	357	357	357	357	315

**Table 6:** Comparison of various evaluation measures for non-COVID class.

Performance measure	VGG16	DenseNet121	MobileNet	Xception	NASNet	EfficientNet
Precision	0.96	0.99	0.94	0.95	0.84	0.63
Recall	1.00	0.96	0.99	0.89	0.96	0.95
*F*1-score	0.98	0.97	0.96	0.92	0.90	0.76
Support	334	334	334	334	334	307

**Table 7:** Comparison of existing system and proposed system.

Models	Existing system	Proposed system
VGG16	79.01%	97.68%
Xception	88.03%	92.47%
DenseNet21	89.96%	97.53%
NASNet	85.05%	89.51%
EfficientNet	93.48%	80.19%

## Data Availability

The data used to support the findings of this study are included in the article.
